The article "Based on UPLC-Q-TOF-MS/MS, Systematic Network Pharmacology, and Molecular Docking to Explore the Potential Mechanism of Fructus Aurantii for Major Depression Disorder" was published in 2021. Journal: Evid Based Complement Alternat Med.

# Based on UPLC-Q-TOF-MS/MS, Systematic Network Pharmacology, and Molecular Docking to Explore the Potential Mechanism of Fructus Aurantii for Major Depression Disorder

**DOI:** 10.1155/2021/6486287

**Published:** 2021-10-08

**Authors:** Yating Xie, Ying Liu, Peng Zheng, Tao Zhang, Xianwen Ye, Minmin Liu, Min Huang, Quan Wan, Jinlian Zhang

**Affiliations:** ^1^School of Pharmacy, Jiangxi University of Chinese Medicine, Nanchang 330004, China; ^2^School of Chinese Material Medica, Beijing University of Chinese Medicine, Beijing 100102, China

## Abstract

**Background:**

Major Depression Disorder (MDD) is a common mental disease that has become one of the world's major medical diseases. Currently, the Fructus Aurantii (FA) has been widely used to treat depression. However, the active substance ingredients and potential mechanisms of the shell antidepression have not yet been clarified.

**Method:**

First, we used ultraperformance liquid chromatography-quadrupole/time-of-flight tandem mass (UPLC-QTOF-MS/MS) technology to identify the chemical composition of the FA. Then, it is predicted for active ingredients, pharmaceutical disease target screening by DiscoveryStudio 2016 (DS), Metascape, and other databases, PPI network diagram, and FC core pathway. Finally, the system network pharmacology results are verified by molecular contact verification.

**Results:**

Forty-six compounds in FA were identified, and twelve active ingredients were determined. Various database information, PPI network analysis of 41 intersections, and 20 core targets including DRD2, MTOR, FASP3, and PIK3P1 were integrated. Finally, the MDD treatment is indicated by molecular docking, and the most relevant potential signal pathway is the PI3K-Akt signaling pathway.

## 1. Introduction

Major Depression Disorder (MDD) is the most common chronic mental disease nowadays, mainly manifested as depression, loss of pleasure, cognitive impairment, panic, lack of initiative, anorexia, insomnia, suicide injury, and other behaviors. Therefore, it is difficult to treat this disease due to its complexity, heterogeneity, and high recurrence [1–4]. Many records related to depression treated using traditional Chinese medicine are available, which divide MDD into six syndrome types: liver depression and spleen deficiency, liver depression and phlegm stagnation, liver depression and qi stagnation, heart and spleen deficiency, heart and kidney disharmony, and qi stagnation and blood stasis [5]. According to the latest report released by the World Health Organization (WHO), there are about 350 million people suffering from MDD in the world, with an average incidence of 4.4%. It is estimated that depression will become the world's largest burden disease by 2030 [6, 7]. At present, the pathogenesis of MDD has not yet been established, and the conventional western medicine uses fluoxetine hydrochloride and sertraline, which are exerting side effects, so it is difficult for them to achieve satisfactory treatment effect. In general, antidepressants cause side effects that ruin the normal daily life, so that patients have poor compliance.

Therefore, in this work, the multicomponent approach used by the traditional Chinese medicine was compared to the traditional treatment of MDD in consideration of the shortcomings of western medicine.

Fructus Aurantii (FA) is the dry immature fruit of the *Citrus Aurantium* L. It often used as a Chinese medicine for regulating qi and used in clinical practice and is one of the components of the most common Chinese medicine prescriptions, including Chaihu Shugan San and Weichang Anwan [8, 9]. The main active ingredients of the FA include flavonoids, coumarins, volatile oils, and alkaloids, which exert an antidepressant effect [10], lower the cholesterol [11], have antitumor effect [12], promote the gastrointestinal power [13], and have other pharmacological activities. Psychological stress due to MDD can lead to gastric emptying and abnormal gastrointestinal hormone levels; FA not only has antidepressant effects, but also promotes the gastrointestinal power by regulating the hypothalamic-pituitary-adrenal axis, alleviating the discomfort caused by MDD [14]. However, the mechanism of action of FA on MDD is not yet clear. Therefore, this study explored the potential mechanism of FA on MDD using UPLC-QTOF-MS/MS, system network pharmacology, and molecular docking (Figure 1).

The FA is mainly produced in the province of Jiangxi, and it is of the highest quality. Therefore, this experiment used FA as raw material, and the chemical composition was determined by UPLC-QTOF-MS/MS. In addition, the active ingredient, disease target, and the action pathway were investigated to obtain the underlined mechanism used by FA on MDD, which was further verified by molecular docking [15–17].

## 2. Materials and Methods

### 2.1. Chemicals, Agents, and Materials

FA was purchased in Yicheng Town, Zhangshu City, Jiangxi Province (Jiangxi, China).

Professor Geifei, who is the head of the Chinese Medicine Resources Discipline Group, at the Jiangxi University of Traditional Chinese Medicine characterized the dry unripe fruit of *Citrus aurantium* L. Twelve pure compounds (purity >98%) such as eriodictyol, 5-demethylnobiletin, naringenin, nobiletin, 3′, 4′, 3, 5, 6, 7, 8-heptamethoxyflavone, auraptene, ferulic acid, umbelliferone, hesperidin, naringin, neohesperidin, and limonin were selected according to the 2015 “*Chinese Pharmacopoeia*” method to process FA and purchased from Sichuan Vicky Biotechnology Co. Ltd. (Sichuan, China). Methanol was purchased from Xilong Scientific Co, Ltd. (Guangdong, China). Acetonitrile (Tedia, USA), formic acid (ACS), and ethanol were purchased from the National Medicine Group Chemical Reagent Co., Ltd. (Shanghai, China). The water used in this work was ultrapure, obtained by the Milli-QB system.

## 3. UPLC-QTOF-MS/MS

### 3.1. Preparation of the Standard and Sample Solutions

The impurities were removed from FA, then it was washed, moisturized, and cut into thin slices, and the broken core was sifted out after drying [18]. FA crude powder (10 g) was precisely weighed and placed in a conical bottle with 100 ml 70% ethanol, thoroughly mixed, socked for 0.5 h, and boiled under reflux for 1.5 h, and the filtrate was collected. In the above methods, 80 mL 70% ethanol and 60 ml 70% ethanol were used. Three filtrates were mixed, and the filtrate was condensed and made into extract. Then, 1 g concrete was weighed and placed in 100 ml methanol to dilute it. Finally, the solution was filtered through a 0.22 mm microporous membrane.

Twelve milligrams of each reference compound (eriodictyol; 5-demethylnobiletin; naringenin; nobiletin; 3′, 4′, 3, 5, 6, 7, 8-heptamethoxyflavone; auraptene; ferulic acid; umbelliferone; hesperidin; naringin; neohesperidin; and limonin) was weighed, transferred to 10 ml volumetric flasks, and diluted with methanol to reach the volumetric mark. The solutions were filtered through a 0.22 *μ*m microporous membrane to obtain the standard solutions.

### 3.2. Ultraperformance Liquid Chromatography-Quadrupole-Time-of-Flight Tandem Mass Conditions

Chemical analysis was conducted on a UPLC- (Nexera X2 LC-30A, Shimadzu Corp., Japan) hybrid triple quadrupole-time-of-flight mass spectrometer (Triple TOF™5600+, AB Sciex, Forster City, FA, USA) connected with an electrospray ionization source (ESI). Acquity UPLC BEH C18 column (2.1 × 100 mm × 1.7 *μ*m) was used to perform the chromatographic separation with a flow rate of 0.3 ml/min at 40°C. A linear gradient program with a mobile phase system including solvent A (100% acetonitrile, v/v) and solvent B (0.01% formic acid in water, v/v) was performed as follows: solvent A at 5% ∼20% for 0.01∼2 min, 20%∼30% for 2∼10 min, 30∼55% for 10∼25 min, 55%∼100% for 25∼30 min, 100% A for 30∼32 min, and 100%∼5% for 0.5 min, with isocratic elution performed at 5% for 2.5 min.

The instrumental setting of Q-TOF-MS/MS was the following: ion source gas 1 (GSI) and gas 2 (GS2) were both set to 60 kPa, curtain gas (CUR) was set to 35 kPa, ion spray voltage floating (ISVF) was set to 5500 V, ion source temperature (TEM) was set at 500°C, collision energy (CE) was set at 45 eV, collision energy spread (CES) was set at 45 ± 10 eV, the declustering potential (DP) was set at 100 V, and nitrogen was used as a nebulizer and auxiliary gas. Samples were analyzed in positive ionization modes with a sFAnnin mass-to-charge (m/z) range from 50 to 1,000. Data were collected in information-dependent acquisition (IDA) mode and analyzed by PeakView®1.2 software (AB Sciex).

### 3.3. Ingredients Identification Analysis

The chemical composition of FA was obtained from existing databases and documents, including TCMSP, SCHINDER, TCMIP, China Knowledge Network, and Geen Medical. The data were sorted out and the FA composition database was established. (+) MS data was imported into PeakView®1.2, “XIC Manager” was used to analyze the 70% ethanol extract of FA, and each chemical composition in the retention time and its corresponding primary and secondary mass spectrum data were obtained. It combined the base peak chart with the reference substance and compared it with the data reported in the relevant references, and the chemical composition was confirmed.

### 3.4. Identification of the Related Targets of FA Components

In this study, the chemical compounds were imported into Discovery Studio 2016 (DS), through “ADMET Descriptors” to screen the active ingredients. The related targets of FA components were obtained from SwissTargetPrediction (https://www.swisstargetprediction.ch/) and Pharmmapper (https://www.lilab-ecust.cn/pharmmapper/).

### 3.5. MDD-Associated Targets Collection

The keyword “depression” was used in the Genecards database (https://www.geneFArds.org/) and Online Mendelian Inheritance in Man (OMIM, https://omim.org/) to identify disease targets associated with MDD.

### 3.6. Construction of the Protein-Protein Interaction Network

VENNY2.1 software (https://bioinfogp.cnb.csic.es/tools/venny/index.html) was used to obtain the overlapping targets between FA-related targets and MDD-related targets. Overlapping targets were imported into the Retrieval of Interacting Genes/Proteins (STRING) 11.0 (https://www.string-db.org/), and the interaction results were saved. The interaction resulting file was added to Cytoscape v3.9.0 software, and the Protein-Protein Interaction (PPI) network was obtained.

### 3.7. Go Function and Genomes (KEGG) Pathway Enrichment Analysis

Metascape is a powerful tool for the analysis of gene function annotation. It applies the bioinformatics analysis method to a large number of genes or proteins, and it uses more than 40 independent databases to annotate genes or proteins, for the enrichment analysis and the construction of the PPI network. WebGestalt was used to perform the enrichment analysis. The software can meet user requirements from different areas, by pathway figure and hierarchical network visualization. Since its release in 2005, it has gradually become one of the most popular software types in the field of biology [19].

Overlapping targets were imported into Metascape (https://www.metascape.org/), “Homo sapiens” was selected as “Organism of interest,” and “Pathway” and “KEGG” were selected as “Functional Database.” Finally, “genome” was selected as the “Select reference set,” and the KEGG pathway analysis was performed.

### 3.8. I-D-G Network Construction

Related files were established as “core ingredients-core targets,” “core ingredients-Secondary targets,” “disease-core targets,” and “disease-Secondary targets.” Then, the files were imported into Cytoscape v3.9.0 to build a “ingredients-disease-gene symbols” network.

### 3.9. Computational Validation of I-T Interactions

The computational software was used to simulate the interaction between active compounds and core targets and to explore the binding ability and binding mode between compounds and targets. Therefore, 12 drug components were selected for the molecular docking with 14 core targets. The PDB format of the target protein was downloaded from the structural bioinformatics protein database (PDB, https://www.rcsb.org/). The protein structure was used to simulate dehydration, hydrogenation, and removal of proteins using DiscoveryStudio2016 (DS) software, and then molecular docking was performed.

## 4. Results

### 4.1. Identification of the Chemical Constituents in FA by UPLC-QTOF-MS/MS

UPLC-QTOF-MS/MS is an analytical technique widely used in drug research, which can perform chromatography and identify fragment ions and cleavage patterns.  Figure 2 represents a (+) ESI-MS mass total ion chromatogram of the FA extract (TIC). A total of 46 compounds were identified using PeakView®1.2 software and literature comparison, including 33 flavonoids, 10 coumarins, 3 limonoids, and other compounds. Twelve ingredients (eriodictyol; 5-demethylnobiletin; naringenin; nobiletin; 3′, 4′, 3, 5, 6, 7, 8-heptamethoxyflavone; auraptene; ferulic acid; umbelliferone, hesperidin; naringin; neohesperidin; limonin) were confirmed by the comparison with the reference substance (Table 1).

### 4.2. Screening of the Active Components in FA

The blood-brain barrier (BBB) is an important structure in the human body to maintain a stable brain environment; thus, lipophilic and water-soluble drugs do not cross easily the BBB, limiting the effect of 95% of drugs on the central nervous system [25]. Depression is a neurological disorder occurring in the central nervous system; thus, the relationship between the ability of antidepressants and the permeability of the BBB is of utmost importance to obtain an effective result.

Forty-six compounds were screened by DS software, and the screening standard used was “ADMET_BBB ≥ −0.3” [26]. Seven active compounds of FA were obtained, such as isomerancin, meranzin, prangenin, bergapten, 5, 6, 7, 4′-tetramethoxyflavone, 3′, 4′, 7, 8-tetramethoxyflavone, and Scutellarein. Scutellarein has a good permeability in the BBB model in vitro, has the ability to improve BBB dysfunction, and treats stroke, Alzheimer's disease, and other central nervous system diseases [27, 28]. Bergapten has extremely high bioavailability, can cross the BBB, protect nerves, and treat brain diseases, and it is a potential candidate as antidepressant drug [29]. However, some compounds not meeting the screening criteria were also chosen in order to comprehensively evaluate MDD treatment. For example, naringin and neohesperidin are the main components of FA according to the 2020 “*China Pharmacopoeia.*” In addition, according to the literature, meranzin hydrate and nobiletin can reduce ROS, MDA, IL-6, and TNF-*α* levels in MDD rats; these compounds can cause anti-inflammatory and antioxidative stress [30]. Naringin can improve the hippocampus mTOR and P70S6K phosphorylation level [31]. Hesperidin can improve CUMS rat behavior by regulating the function of the hypothalamic-pituitary-adrenal (HPA) axis [32]. Although these compounds do not satisfy the screening criteria of crossing the BBB, some studies showed their biological activity; thus, these 5 compounds were also used as candidate active components. Finally, 12 compounds were chosen as active ingredients (Table 2).

### 4.3. Acquisition of the Related Targets of FA Components

All the targets of the compounds in FA were collected from the SwissTargetPrediction software and Pharmmapper software. A total of 827 FA-related targets were obtained after the removal of the repeated targets.

### 4.4. Identification of the MDD-Associated Targets

The screening standard used was “Relevance score>10” [33], which allowed obtaining 71 and 189 MDD-related targets by Genecard database and OMIM database, respectively. A total of 238 known MDD-related targets were collected after the removal of the redundant information.

### 4.5. PPI Network Analysis

The disease targets and composition targets were combined and imported into Venny2.1 software, and 41 overlapping targets were obtained by the Venny diagram (Figure 3(a)) and PPI network (Figure 3(c)). The PPI network diagram was visualized by the Cytoscape software for a further analysis (Figure 3(b)). The results showed that NCS1 did not intersect with other targets. “Degree” could allow the evaluation of the effect to each target to a certain extent; thus, the median value of “degree” was used as a screening condition [34], and degree was ranked as a core target (Figure 3(d)). For example, DRD2, FASP3, and PIK3P1 could be important research targets for the treatment of MDD with FA.

### 4.6. Analysis of the Go and KEGG Pathway Enrichment

WebGestalt and Metascape were used to perform Go function and KEGG pathway enrichment analysis on 20 core targets. The results showed the involvement of 12 Biological Processes (BP), 16 Cellular Components (CC), and 13 Molecular Functions (MF). BP was related to cell communication, response to stimulus, and biological regulation, CC was related to membrane, cell projection, and endomembrane system, and MF was related to protein binding, molecular transducer activity, and ion binding (Figure 4(a)).

There is a close relationship between the core target and the signaling pathway. The screening results with “value of enrichment ratio” resulted in 10 pathways, including EGFR tyrosine kinase inhibitor resistance (hsa04080), ErbB signaling pathway (hsa04072), thyroid hormone signaling pathway (hsa04919), PI3K-Akt signaling pathway (hsa04151), and neuroactive ligand-receptor interaction (hsa04722). Some antidepressants exert a therapeutic effect through the ErbB signaling pathway and often induce the downregulation of NRG1/ErbB4; thus, our hypothesis was that antidepressants could play a role through this channel [35]. Therefore, the above pathways were obtained by screening, providing a direction in the research of a new mechanism of action of FA.

### 4.7. I-D-G Network Analysis

Cytoscape v3.9.0 software was used to build an “ingredients-disease-gene symbols” network, as shown in Figure 5, in which the pink node represented the common targets, the twelve magenta nodes represented the core ingredients of FA, and the 20 green nodes represented the core gene symbols between FA and MDD. This result revealed that FA could play a role in the treatment of MDD through multiple targets.

Cytoscape software analysis revealed that the values of C4 (isomerancin, degree = 7), C1 (hesperidin, degree = 6), C5 (meranzin, degree = 6), C2 (naringin, degree = 5), and C7 (prangenin, degree = 5) were at the top of the list, meaning that these compounds could be the core components of FA effective in the treatment of MDD.

### 4.8. Computational Validation of I-T Interactions

The binding ability of the receptor to the ligand is closely related to the molecular docking score. The higher the score, the stronger the binding ability of the receptor. The docking scoring results showed that most of the receptors had good binding ability to the ligands except ABL1 and FASP3 genes, which had low docking scores (Table 3). Therefore, the two gene symbols ABL1 and FASP3 were removed during the building of the heat map.  Figure 6(a) shows that the better the color, the higher the docking score. Our results revealed that neohesperidin, naringin, and hesperidin have a high binding ability with DRD4 and mTOR.

Based on these data, we found that the interaction between each component and the core target is the basis of biological activity. Therefore, FA in the treatment of MDD is a complex process among a series of multitargets and multicomponents.

## 5. Discussion

MDD is a common mental disease that has become one of the world's major diseases, resulting in the change of the quality of life and work ability. The number of patients increases year by year. At present, most of the patients suffering from clinical depression are treated by the western medicine, which commonly use selective serotonin reuptake inhibitors (fluoxetine and paroxetine) and serotonin and norepinephrine reuptake inhibitors (venlafaxine and duloxetine). However, many problems are associated with the use of the western medicine, such as high recurrence rate, poor tolerance, and adverse reactions. The treatment using traditional Chinese medicine is gradual, and the existing research results show that the curative effect of the Chinese medicine does not differ significantly from that of the western medicine. Nevertheless, the Chinese medicine has a faster effect, less adverse reactions, and more benefits. Therefore, the research on MDD of traditional Chinese medicine has been more intense and fruitful in recent years.

FA is one of the commonly used medicinal compounds, which is widely used to cure gastrointestinal diseases. Previous studies showed that MDD often leads to gastrointestinal dysfunction, and the FA extract can regulate the HPA axis [36] and neuroprotection [37], regulate gastrointestinal hormones [38], and can participate in regulating monoamine-based syndrome systems [39]. However, the potential mechanism used by FA to cure depression is unknown. This work used network pharmacological methods, detected the active ingredients, targets, and passage, and combined them to obtain the potential mechanism of action of FA on MDD.

UPLC-Q-TOF-MS/MS technology was used to identify FA chemical components. Then, the combination of the literature with the related software resulted in a selection of 12 main active ingredients. Finally, the overlapping target was used to perform the PPI network analysis. DRD2, DRD4, OPRM1, and mTOR were the most relevant targets for the treatment of MDD by FA. DRD2 is divided into two subtypes, D2S and D2L [40], it is a target of many antipsychotic drugs, and its down- or upregulation is closely associate with MDD [41]. mTOR is a receptor serine/threonine kinase, and in its activated, phosphorylated form can regulate the nerves and promote topical protein synthesis, thereby further promoting the synaptic formation [42, 43]. A study found that hesperidin exerted an antidepressant effect by activating the hippocampus mTOR pathway [44]. Interestingly, neohesperidin, naringin, and hesperidin were the key components of FA involved in the treatment of MDD, as shown by the hot map. For example, DRD2 and mTOR had a good molecular binding ability than forneohesperidin and hesperidin. Therefore, our hypothesis was that the above ingredients and targets might represent the key elements on the role of FA as antidepressant.

Metascap was used to perform the pathway analysis on 20 core targets. The results showed that FA mainly activates and regulates PI3K-Akt signaling pathway (hsa04151). EGFR tyrosine kinase inhibitor resistance (hsa04080) and ErbB signaling pathway (hsa04072) exert pharmacological effects. The feature to pay attention to is PI3K-Akt signaling pathway, Akt is upstream of the mTOR signaling pathway, and the phosphorylated form can activate the mTOR signaling pathway. Key targets for PI3K/Akt signaling pathway influence the glutamic acid system function, hippocampal neuron apoptosis, and mitochondrial function involved in MDD. Many studies show the main role of TCM as an antidepressant by acting on the PI3K/Akt/mTOR signaling pathway. Caihujialong Tang increases the expression and activity of PI3K in the rat hippocampus to protect neurons, thus exerting an antidepressant effect [45]. Jiaotai Wan regulates PI3K/AKT/mTOR signaling pathway related proteins to improve depression and reverse behavioral changes in rats [46]. The above evidence generated the hypothesis that FA is effective by acting on AKT, PI3K, and mTOR protein expression.

FA in China is often used as a hydraulic medicine, commonly used to cure gastrointestinal diseases, but the literature does not give any explanation regarding its therapeutic effects on MDD, such as the mitigation of diarrhea caused by MDD. Therefore, our results by UPLC-Q-TOF-MS/MS technology and system pharmacology revealed a potential mechanism of FA to treat MDD, providing a reference for the development and use of antidepressants.

## Figures and Tables

**Figure 1:** Based on systems pharmacology strategy to study the mechanism of FA in treatment of MDD.

**Figure 2:** The (+) ESI-MS mass total ion chromatogram (TICs) of the FA by UPLC/Q-TOF-MS/MS.

**Figure 3:** (a) Venn diagram of related targets of Aurantii Fructus (FA) and Major Depressive Disorder (MDD). (b) PPI network of overlapping targets between drug and disease. The more the color, the higher the value. (c) PPI network. (d) Bar plot of the 20 core targets. The *x*-axis represents the degree. The *y*-axis represents the target protein.

**Figure 4:** (a) Bar plot of the GO function enrichment of core targets. Red represents the Biological Process (BP). Blue represents the Cellular Component (CC). Green represents the Molecular Function (MF). (b) Bubble chart of KEGG enrichment of core targets. The *x*-axis represents the ratio enrichment. The *y*-axis represents the pathway.

**Figure 5:** The I-D-G network.

**Figure 6:** (a) Heatmap of I-G docking scores. (b) 3D diagram of naringin-DRD4 and naringin-mTOR.

**Table 1:** Identification of chemical constituents of FA immaturus ethanol extract.

No	Molecular formula	Extraction mass (Da)	Error (ppm)	tR/(min)	Identity	Classification	Ref.
1	C_27_H_30_O_15_	511.1658	2.8	3.73	Lonicerin	Flavonoid	[20]
2	C_15_H_12_O_6_	289.0707	0.2	4.98	Eriodictyol	Coumarin	[21]
3	C_22_H_24_O_9_	433.1493	1.6	20.45	3′,4′,3,5,6,7,8-Heptamethoxyflavone	Flavonoid	[22]
4	C_27_H_32_O_15_	597.1814	2.3	4.99	Neoeriocitrin	Flavonoid	[20]
5	C_27_H_32_O_15_	597.1814	2.3	4.7	Eriocitrin	Flavonoid	[20]
6	C_10_H_10_O_4_	195.0652	−2.8	5.37	Ferulic acid	Total phenolic acids	[20]
7	C_16_H_14_0_6_	303.0863	0.6	6.88	Hesperetin	Flavonoid	[21]
8	C_27_H_32_O_14_	581.1865	2.4	5.67	Narirutin	Flavonoid	[21]
9	C_15_H_12_O_5_	273.0758	−1	12.04	Naringenin	Flavonoid	[21]
10	C_21_H_22_O_10_	435.1286	1.2	6.07	Naringenin-7-O-glucoside	Flavonoid	[20]
11	C_22_H_24_O_11_	465.1391	0.8	6.87	Hesperetin-7-O-glucoside	Flavonoid	[21]
12	C_28_H_34_O_15_	611.1971	1.6	6.42	Hesperidin	Flavonoid	[20]
13	C_27_H_32_O_14_	581.1865	2.4	6.06	Naringin	Flavonoid	[23]
14	C_28_H_34_O_15_	611.1971	1.6	6.87	Neohesperidin	Flavonoid	[23]
15	C_22_H_24_O_11_	465.1391	0.8	7.24	Eriodictiol-7-O-glucoside	Flavonoid	[21]
16	C_15_H_16_O_4_	261.1121	−0.9	16.22	Isomerancin	Coumarin	[20]
17	C_15_H_16_O_4_	261.1121	−0.9	8.22	Meranzin	Coumarin	[20]
18	C_15_H_18_O_5_	279.1227	−0.1	8.23	Meranzin hydrate	Coumarin	[20]
19	C_11_H_6_O_4_	203.0339	−2.7	9.36	Xanthotoxol	Coumarin	[20]
20	C_26_H_27_O_14_	564.1474	2.6	9.86	Isonaringin	Flavonoid	[20]
21	C_16_H_14_O_5_	287.0914	−0.8	10.45	Prangenin	Coumarin	[21]
22	C_16_H_14_O_5_	287.0914	−0.8	10.47	Isosakuranetin	Flavonoid	[21]
23	C_28_H_34_O_14_	595.2021	1.7	6.88	Poncirin (isosakuranetin-7-O-neohesperidoside)	Flavonoid	[21]
24	C_28_H_34_O_14_	595.2021	1.7	8.22	Neoponcirin	Flavonoid	[21]
25	C_28_H_34_O_14_	595.2021	1.7	9.85	Isosakuranetin-7-O-rutinoside	Flavonoid	[21]
26	C_28_H_34_O_14_	595.2021	1.7	5.89	Poncirin	Flavonoid	[20]
27	C_18_H_16_O_6_	329.102	0.3	11.53	4′-Hydroxy-5,6,7-trimethoxyflavone	Flavonoid	[22]
28	C_12_H_8_O_4_	217.0495	−2.3	14.77	Bergapten	Coumarin	[20]
29	C_19_H_24_O_5_	333.1697	0.5	14.93	Marmin	Coumarin	[20]
30	C_19_H_18_O_6_	343.1176	−0.5	16.98	5,7,8,4′-Tetramethoxyflavone	Flavonoid	[22]
31	C_19_H_18_O_6_	343.1176	−0.5	16.99	5,6,7,4′-Tetramethoxyflavone	Flavonoid	[22]
32	C_19_H_18_O_6_	343.1176	−0.5	19.08	3′, 4′,7,8-Tetramethoxyflavone	Flavonoid	[22]
33	C_19_H_18_O_6_	343.1176	−0.5	11.08	Scutellarein	Flavonoid	[21]
34	C_21_H_22_O_8_	403.1387	0.6	19.04	3,5,7,8,3′, 4′-Hexamethoxyflavone	Flavonoid	[22]
35	C_21_H_22_O_8_	403.1387	0.6	19.05	Nobiletin	Flavonoid	[20]
36	C_28_H_34_O_9_	515.2276	1	19.75	Nomilin	Limonoid	[22]
37	C_20_H_20_O_7_	373.1282	0.7	15.04	5,7,8,3′,4′-Pentamethoxyflavone	Flavonoid	[22]
38	C_20_H_20_O_7_	373.1282	0.7	16.72	Auranetin	Flavonoid	[21]
39	C_20_H_20_O_7_	373.1282	0.7	21.15	Tangeretin	Flavonoid	[23]
40	C_20_H_20_O_7_	373.1282	0.7	16.97	Sinensetin	Flavonoid	[20]
41	C_20_H_20_O_7_	373.1282	0.7	16.72	Isosinensetin	Flavonoid	[21]
42	C_21_H_22_O_9_	419.1337	1.1	21.27	Natsudaidain	Flavonoid	[20]
43	C_20_H_20_O_8_	389.1231	0.2	[23].07	5-Demethylnobiletin	Flavonoid	[22]
44	C_9_H_6_O_3_	163.039	−4.1	5.33	Umbelliferone	Coumarin	[20]
45	C_19_H_22_O_3_	299.1642	−0.3	29.63	Auraptene	Coumarin	[24]
46	C_26_H_30_O_8_	471.2013	−4	17.47	Limonin	Limonoid	[22]

**Table 2:** Absorption parameters of 12 FA components.

No	Component	Molecular formula	BBB
C1	Hesperidin	C_28_H_34_O_15_	ND
C2	Naringin	C_27_H_32_O_14_	ND
C3	Neohesperidin	C_28_H_34_O_15_	ND
C4	Isomerancin	C_15_H_16_O_4_	−0.126
C5	Meranzin	C_15_H_16_O_4_	−0.098
C6	Meranzin hydrate	C_15_H_18_O_5_	−0.852
C7	Prangenin	C_16_H_14_O_5_	−0.282
C8	Bergapten	C_12_H_8_O_4_	−0.233
C9	5,6,7,4′-Tetramethoxyflavone	C_19_H_18_O_6_	−0.185
C10	3′,4′,7,8-Tetramethoxyflavone	C_19_H_18_O_6_	−0.185
C11	Scutellarein	C_19_H_18_O_6_	−0.185
C12	Nobiletin	C_21_H_22_O_8_	−0.478

**Table 3:** DRD docking with the component score.

No	Component	Score
C2	Naringin	186.427
C3	Neohesperidin	178.642
C1	Hesperidin	144.394
C11	Scutellarein	111.055
C10	3′, 4′, 7, 8-Tetramethoxyflavone	109.533
C7	Prangenin	107.563
C4	Isomerancin	103.292
C5	Meranzin	100.242
C6	Meranzin hydrate	100.109
C9	5, 6, 7, 4′-Tetramethoxyflavone	91.912
C8	Bergapten	87.6184
C12	Nobiletin	77.2802

## Data Availability

The data used to support the findings of this study are included within the article.
